# Significance of Circulating Tumor Cells in Nonsmall-Cell Lung Cancer Patients: Prognosis, Chemotherapy Efficacy, and Survival

This article has been retracted.

**DOI:** 10.1155/2021/2680526

**Published:** 2021-11-09

**Authors:** Jianpeng Li

**Affiliations:** Department of Oncology People's Hospital of Xintai City, Xintai Hospital Affiliated to Shandong First Medical University, No. 1329 Xinpu Road, Xintai 271200, Shandong, China

## Abstract

**Introduction:**

We aimed to evaluate whether circulating tumor cells (CTCs) were the prognostic indicator responsible for chemotherapy and survival of NSCLC patients.

**Methods:**

Between January 2013 and September 2017, CTCs in the peripheral blood of histologically confirmed stages III and IV NSCLC patients were collected. Blood specimens were obtained on the first day of treatment, chemotherapy 2 and 4 cycles, or targeted therapy 1 and 2 months for CTCs detection. The positive CTC status was defined as one or more CTCs per 7.5 ml.

**Results:**

100 patients were enrolled, of which 48 patients (48%) were identified to be CTC positive at baseline. A higher CTC-positive rate was observed in stage IV NSCLC patients than stage III patients (69% vs. 40%, *P*=0.015). CTC cluster was significantly correlated with disease control rate. Based on the baseline CTC number, patients were divided into low CTC levels (<4 CTCs, LL) and high CTC levels (≥4 CTCs, HL). There was clinically significant shorter median OS and OS (overall survival) and PFS (progression-free survival) in HL group patients (*P* < 0.001).

**Conclusions:**

The positive association between the CTC number and survival suggested that the baseline CTC number and changes during treatment might be the prognostic information of response rate and overall survival in Chinese patients suffering stage III/IV NSCLC.

## 1. Introduction

Lung cancer owns the highest mortality of all cancers. Nonsmall-cell lung cancers (NSCLCs) as a subtype of lung cancer account for about 85% of cell lung cancers [1, 2]. NSCLC is associated with a poor survival rate for delayed diagnosis [1]. Thus, the identification of biomarkers or indicators for early detection and prognosis prediction was focused on.

Circulating tumor cells (CTCs) that existed in the blood samples are considered to be detached from the primary tumor tissues consistently [3–5]. CTCs are characteristic by positive expression of cytokeratins (CKs) 8/18 and/or 19 and EpCAM (epithelial cell markers) and negative expression of CD45 [6–8]. Circulating CTCs also exhibit metastatic character [9, 10]. CTCs are supposed to be a risk factor for metastasis [11]. CTCs have been applied as the noninvasive method to assess cancer properties quantitatively and qualitatively [12–14].

Recently, CTCs identification provided the evidence for the hypothesis of the diffusion of cancer cells via vascular transmission [15]. It is reported that CTCs are responsible for the aggressiveness property of advanced cancers, contributing to the tumor cell metastasis from primary site to distant site through blood circulation in NSCLC [4, 16]. However, the prognostic impact of CTCs on NSCLCs has not been fully understood [5, 17].

In this study, the predictive prognosis value of CTCs in NSCLC was evaluated, and the risk factor of other factors on the survival of NSCLCs was combinatively evaluated. We attempted to further improve the knowledge of the biological characteristics of CTCs.

## 2. Methods

### 2.1. Subjects' Selection Criteria

Approval was obtained from the local ethical board, and the procedures of studies involved with human subjects were confirmed to the principles of the Declaration of Helsinki. All enrolled patients had signed the written informed consent. Between January 2013 and September 2017, NSCLC patients diagnosed at stages III and IV were enrolled, based on CT, MRI, and histopathologic examination.

Inclusion criteria were measurable NSCLC, and Eastern Cooperative Oncology Group score of 0–2. All NSCLC patients were treatment-naive. Patients with EGFR mutation accepted EGFR-TKIs targeted therapy until disease progression. The other patients received chemotherapy with 4 cycles of intravenous injection of docetaxel 100 mg/m^2^ on days 1 and 8 or pemetrexed 500 mg/m^2^ on day 1 and IV cisplatin 25 mg/m^2^ on days 1, 2, and 3 for consecutive 3 weeks.

### 2.2. CTC Detection and Identification

Before starting treatment, the blood specimens of included patients were collected for the baseline CTCs evaluation. After treatment, CTCs were detected on the first day, chemotherapy 2 and 4 cycles, or targeted therapy 1 and 2 months. The first 6 ml of blood was discarded to avoid epithelial contamination caused by skin puncture. To avoid epithelial contamination, 4 ml of median vein blood was collected in the ADC anticoagulative tube after discarding the first 6 ml of blood samples.

Negative enrichment of immune magnetic beads and FISH were used to detect CTCs. Enriched cells were characterized by fluorescence in situ hybridization labeled with centromere probe 8 (CEP8) and Alexa Fluor 594-anti-CD45 IgG (Bioorth Biotechnology). Nuclear staining was achieved by DAPI (Jiuling Chemical Co., Ltd.) containing an antifade mounting medium. A cell with CKpos/EpCAMpos/CD45neg and a DAPIpos nucleus was defined as a CTC according to FDA-approved recommendation [7]. A CTC cluster was considered to be an aggregate with ≥2 CTCs [2].

### 2.3. Statistical Analysis

At baseline, the clinical information of specimens was collected and analyzed based on the blinded method. After treatment, the physical indexes and blood chemistry parameters were tested once a week, and a CT scan was performed after every two cycles of chemotherapy. In the first 2 years of the follow-up period, physical examination and a thoracic CT were performed every 3 months, and then, the follow-up examinations were performed every 6 months. Patients with suspected recurrence were subjected to other imaging examinations. The Response Evaluation Criteria in Solid Tumors (RECIST) version 1.0 was executed to evaluate the objective response rate (ORR) as complete response (CR), partial response (PR), stable disease (SD), or progressive disease (PD). The outcomes above were assessed on the first day of treatment. SPSS 18.0 was executed for statistical analysis. The prognostic value of CTCs on OS and PFS was evaluated by the K-M method. The effect of CTC and other influence factors on OS and PFS were assessed by the Cox regression model. *P* < 0.05 indicated a statistical significance.

## 3. Results

### 3.1. Prognostic Significance of Circulating Biomarkers

Between January 2013 and September 2017, 102 patients were enrolled, and two patients with no CTC were excluded. The baseline clinical information of eligible patients is given in Table 1. Total 100 patients (male: 65, female: 35) with median age of 67 years (ranged 44.2–76.4) were included, among which 47 were squamous cell cancer and 49 were adenocarcinoma. There were 44 stage III patients and 56 stage IV patients. In addition, 43 patients were present with a smoking history.

### 3.2. Relationships between CTC Counts and Clinical Information

Positive CTC status (2 CTCs/4 ml blood, ranged 0–97) were found in 48 patients (48%) at baseline. CTCs counts were increased in patients from stages III to IV (*P* < 0.001). A higher CTC-positive rate was observed in stage IV NSCLC patients than stage III patients (69% vs. 40%, *P*=0.015). In addition to this, there were no significant correlations found between CTC status and other clinical parameters, such as age, sex, smoking history, and NSCLC histologic subtypes (Table 2).

### 3.3. Relationship of CTCs to Response to Treatment

During the follow-up, all the patients were subjected to an imaging monitor study assessed by RECIST. The disease control rate (DCR) after 2 cycles of chemotherapy or 4 weeks of targeted therapy was 58% (6 CR, 16 PR and 36 SD), while 42 patients had PD. The average CTC counts of patients with DCR was relatively lower than that in patients with PD. After four cycles of chemotherapy or 8 weeks of targeted therapy, 36 patients had SD, 6 had CR, 16 had PR, and 42 had PD. Significant correlations were found between CTC status and DCR (Table 3). Additionally, compared with baseline, the CTC counts were decreased in 57 patients, increased in 14 patients, and remained stable in 29 patients (Table 4).

### 3.4. Relationship between CTC Counts and Survival

According to baseline CTC number, patients were divided into low CTC level (<4 CTCs, LL) and high CTC level (≥4 CTCs, HL) groups, followed by CTC univariate analysis. CTC-positive patients were present with shorter median OS. The median follow-up time of patients was 17.0 months (range, 3–36 months), the median survival time (MST) was 9.1 months (95% CI: 8.3–9.9 months) in the LL group, and 6.8 months (95% CI: 6.1–7.4 months) in the HL group (*P* < 0.001, Figure 1). Overall, 1-year survival rates were 71.8% (95% CI: 64.6%–79%) and 41.2% (95% CI: 29.3%–53.1%) in the LL and HL groups, respectively. Clinically, a significant difference was present in OS between high and low CRC groups. Moreover, a shorter median of PFS was observed in patients with favorable CTC counts. Patients in the LL group showed higher PFS (median 5.6 months, 95% CI: 2.9–8.2) than that in the HL group (median 4.2 months, 95% CI: 3.8–4.6) (*P* < 0.001, Figure 2).

## 4. Discussion

The current study showed that the CTC counts at baseline had significant correlations between CTC cluster and DCR. The declined CTC count in patients after 4 cycles of chemotherapy was a predictive factor for DCR. Moreover, patients with favorable CTC count at baseline were closely related to the shorter OS and PFS.

In the current study, 48% of patients with metastatic NSCLC were present with positive CTC in blood samples. Tanaka et al. [18] and Hirose et al. [19] have suggested that patients could be diagnosed with lung cancer with the cutoff value for CTC count as one per 7.5 ml of blood. The positive CTC status took account for 30% and 36.4% of lung cancer patients with one and more CTCs per 7.5 ml of blood, respectively. In fact, the cutoff point of 1 or 2 CTC in lung cancer diagnosis was widely recommended by other researchers. The study of Krebs et al. [20] proposed a positive CTC status as one CTC per 7.5 ml peripheral blood and identified that the baseline CTC number of 2 was found in 32% of patients with metastatic disease. These results are consistent with our findings.

Currently, the predictive role of CTCs on chemotherapy response in NSCLC patients has been rarely investigated [20–23]. Physicians need to make individual treatment management based on the response of patients to cytotoxic chemotherapy. Our data showed that patients with positive CTC status at baseline exhibited a higher rate of progressive disease responses to progressive disease than patients with negative CTC status. The study of Hirose et al. [19] evaluated CTC status in NSCLC patients with combination chemotherapy of gemcitabine and carboplatin. They reported that poor prognosis was found in patients with 5 CTCs postchemotherapy, compared with those with CTCs less than 5. The result is identical to our study. The patients with negative CTC status at baseline remained the same CTC status after the second chemotherapy cycle. The changes in CTC levels before and after the second cycle of chemotherapy were significantly correlated with the progressive disease rate [24, 25]. In addition to this, the study of Muinelo-Romay et al. [26] has supposed CTC count as the prognosis biomarker for chemotherapy response.

In demonstrating that CTCs were predictive of survival, we found that patients with high CTC levels (≥4 CTCs) had a remarkably shorter OS than those with CTCs <4. The study of Hofman et al. [15] indicated that CTC level (≥ 50 CTCs) predicted shorter OS and PFS in NSCLC. But few patients have so high CTCs. So, the relationship with the proper CTC level with OS still needs to be defined. Recently, Zhang et al. [27] indicated that the PFS and OS values were significantly different for patients with the CTC level (<8 CTCs) and CTC level (≥8 CTCs). But in the study, only 46 patients were enrolled, including 39 patients in the low CTCs group and only seven patients in the high (≥8) CTCs group. The effect of a small sample size in a high CTCs group on results should be interpreted. Moreover, combined with the previous studies, we were able to identify a proper CTC cutoff (<4 CTCs), presenting fewer CTCs amount particularly having longer survival.

In conclusion, we demonstrated that the CTC level showed a predictive value for DCR and the response rate to chemotherapy. Moreover, CTC levels have a significant connection with OS and PFS. Thus, CTCs could be proposed as an important prognostic factor for chemotherapy efficacy in NSCLC patients.

## Figures and Tables

**Figure 1:** Kaplan–Meier curve for overall survival (OS) according to the levels of the circulating tumor cells (CTCs).

**Figure 2:** Kaplan–Meier curve for progression-free survival (PFS) according to the levels of the circulating tumor cells (CTCs).

**Table 1:** Patient demographics.

Characteristic	No.
Age	
≤59	41
>59	59

Sex	
Male	65
Female	35

Smoking status	
Former smoker	53
Never smoker	47

Histology	
Squamous cell cancer	49
Adenocarcinoma	47
Poorly differentiated	4

Tumor stage	
III	44
IV	56

**Table 2:** Prevalence of CTCs association with clinical characteristics.

Characteristic	No. of patients		*P*
	No. of positive	No. of negative	
Age			
≤59	18 (44%)	23 (56%)	0.863
>59	30 (51%)	29 (49%)	

Sex			
Male	35 (54%)	30 (46%)	0.409
Female	21 (60%)	14 (40%)	

Smoking status			
Former smoker	26 (49%)	27 (51%)	0.345
Never smoker	20 (43%)	27 (56%)	

Histology			
Squamous cell cancer	26 (53%)	23 (46%)	0.392
Adenocarcinoma	22 (47%)	25 (53%)	
Poorly differentiated	2 (50%)	2 (50%)	

Tumor stage			
III	18 (41%)	26 (59%)	0.015
IV	39 (70%)	17 (30%)	

**Table 3:** Response rates according to the levels of CTCs.

Response	No. of patients			*P*
	Positive	Negative	Total	
Disease control rate	22 (38%)	36 (62%)	58	<0.001
Progressive disease	23 (64%)	13 (36%)	36	

**Table 4:** Response rates association with the changes of CTCs.

Changes	Response				Total	*P*
	CR	PR	SD	PD		
Up	0 (0%)	1 (2%)	6 (1.5%)	32 (82%)	39	<0.001
Stable	2 (13%)	2 (13%)	9 (60%)	2 (13%)	15	
Down	4 (9%)	13 (28%)	21 (46%)	8 (17%)	46	
Total	6 (6%)	16 (16%)	36 (36%)	42 (42%)	100	

## Data Availability

The simulation experiment data used to support the findings of this study are available from the corresponding author upon request.
